RETRACTED

# Mesenchymal Stem Cell Exosomal miR-146a Mediates the Regulation of the TLR4/MyD88/NF-*κ*B Signaling Pathway in Inflammation due to Diabetic Retinopathy

**DOI:** 10.1155/2022/3864863

**Published:** 2022-06-18

**Authors:** Cao Gu, Hongjun Zhang, Shaofei Zhao, Daotong He, Yu Gao

**Affiliations:** ^1^Department of Ophthalmology, Changhai Hospital Affiliated to Navy Medical University, Shanghai 200433, China; ^2^Department of Ophthalmology, Minhang Branch of Zhongshan Hospital Affiliated to Fudan University, Shanghai 201100, China

## Abstract

Diabetic retinopathy (DR) is the main cause of vision loss in diabetic patients, which cannot be completely resolved by typical blood sugar control. Inflammation influences the development of DR, so reducing the inflammatory response in DR patients is crucial to the prevention of DR. Therefore, we explored the regulatory effect of bone marrow mesenchymal stem cell (BMSC) exosomes on inflammation in DR mice. In order to analyze the mechanism of action, we used BMSC exosomal miR-146a to treat microglias in DR mice to observe cellular changes and expression of inflammatory factors. It was found that BMSC exosomal miR-146a reduced the levels of proliferating cell antigen and B-cell lymphoma-2 in microglias of DR mice and increased Bcl-2-related X with cysteine aspartic protease-3. By analyzing the expression of inflammatory factors, we found that BMSC exosomal miR-146a reduced the levels of TNF-*α*, IL-1*β*, and IL-6, which suggested that miR-146a can alleviate inflammation in DR mice. Further exploration found that miR-146a reduced the activity of TLR4 and increased the activity of MyD88 and NF-*κ*B. Furthermore, the overexpression of TLR4 reversed the effects of miR-146a on the proliferation, apoptosis, and inflammation of microglias. Our study demonstrated that BMSC exosomal miR-146a can regulate the inflammatory response of DR by mediating the TLR4/MyD88/NF-*κ*B pathway, providing an experimental basis for the prevention and treatment of DR.

## 1. Introduction

Diabetic retinopathy (DR) is a common ocular complication caused by diabetes. Patients with DR have no obvious clinical symptoms early on, but vision is impaired when the disease progresses to a more severe stage [1], during which patients experience tenderness of the eyeball, blurred, or loss of vision and floaters [2, 3]. Failure to get timely and effective treatment can result in blindness in both eyes. Conventional DR therapy aims to control blood sugar with drugs, prevent further deterioration of the disease, and improve vision and metabolic function of the body [4]. However, some clinical practices show that despite achieving effective blood sugar control, some patients still progress to a more severe stage of DR. Therefore, identifying new treatment strategies to prevent or slow down disease progression of DR has become a focus of attention. DR is a microvascular complication of diabetes, which is characterized by the loss of retinal capillary pericytes and increased vascular permeability [5]. Studies have confirmed that inflammation promotes the development of DR [6–8]. Chronic inflammation can cause dysfunction of the retinal endothelial cells, reduce pericytes, and increase vascular permeability, which contribute to the progression of DR [7]. Microglias are the main immune cells of the central nervous system. In healthy retinas, microglias are mainly distributed in the inner layer of the retina [9], while in pathological conditions, a large number of activated microglias can be found in the space between the outer nuclear and subretinal layers [10]. Long-term activation and continuous proliferation of microglias can cause massive secretions of inflammatory cytokines, activation of the apoptotic protein Caspase, and apoptosis of retinal nerve cells, leading to the development of DR [11, 12]. Therefore, effective inhibition of microglial activation and proliferation is crucial for reducing chronic inflammation in patients with DR.

RETRACTED

In recent years, stem cell therapy has provided new approaches for clinical treatment of DR. Bone marrow mesenchymal stem cells (BMSCs) are a subgroup of mammalian bone marrow stromal cells with a multidirectional differentiation potential. Studies have confirmed that BMSCs can promote the secretion of neurotrophic factors, increase the growth rate of nerve fibers, and inhibit inflammation [13]. miR-146a is a single-stranded noncoding small RNA that regulates gene expression by binding to target mRNAs. As an important innate immune signal regulator, miR-146a is involved in the immune response process of various autoimmune and infectious diseases [14]. Exosomes are nanoscale particles that can effectively deliver miRNA to recipient cells. Studies have shown that BMSCs modulate tumor microenvironment by secreting exosomal miRNAs, thereby affecting the biological behavior of tumor cells [15]. The toll-like receptor 4 (TLR4)/myeloid differentiation factor 88 (MyD88)/nuclear transcription factor-*κ*B (NF-*κ*B) signaling pathway is shown to be closely related to the body's immune response [16]. TLR4 transmits signals through the MyD88 signaling pathway mediated by the MyD88 adaptor protein, which binds to phosphorylated adaptor factors and travels downstream to the NF-*κ*B pathway, leading to the activation of transcription factors [17]. Studies have reported that lipase (LPS) can mediate the production of TNF-*α*, IL-6, and IL-8 in patients with liver cancer via the TLR4/MyD88/NF-*κ*B signaling pathway and activate the cyclooxygenase-2/prostaglandin signal axis, thus regulating the proliferation of liver cancer cells [18]. The activation of the TLR4/MyD88/NF-*κ*B pathway can not only improve antitumor immunity but may also cause tumor immune surveillance and promote tumor development [19]. Therefore, this study is aimed at studying the effect of BMSC exosomal miR-146a on microglia-mediated inflammation and explore whether its mechanism of action is associated with the TLR4/MyD88/NF-*κ*B signaling pathway.

RETRACTED

## 2. Materials and Methods

### 2.1. Animals, Reagents, and Instruments

The experimental mice, 6-8 weeks old male C57BL/C, were provided by the Guangxi Animal Experiment Center. Streptozotocin was provided by Dalian Meilun Biotechnology Co., Ltd. Fetal bovine serum was supplied by Hangzhou Sijiqing Bioengineering Materials Co., Ltd. Dulbecco's modified Eagle medium (DMEM) was provided by Hycilne, USA. 3-(4, 5-Dimethylthiazole-2)-2, 5-diphenyl-tetrazolium bromide (MTT) and dimethyl sulfoxide (DMSO) were both supplied by Sigma-Aldrich. The high-speed centrifuge was provided by Hunan Xiangyi Centrifuge Co., Ltd. The flow cytometer was provided by the American BD Company. The enzyme-linked immunosorbent assay kit was provided by Rapibio Lab, USA.

This study was approved by the institutional animal care and use committee of Changhai Hospital Affiliated to Navy Medical University, Shanghai, China, and was conducted in strict accordance with the guidelines of the Association for Research in Vision and Ophthalmology (ARVO) for the use of animals.

### 2.2. Isolation, Culture, and Identification of BMSCs

The experimental mice were sacrificed using the whole bone marrow method and placed in 75% alcohol for 10 min. On a sterile operating table, the lower limb skin of the mouse was cut with sterile scissors, and the thigh and calf muscles were separated to fully expose the tibia and fibula of both lower limbs. The hip and knee joints were severed, and the tibia and fibula were removed and rinsed with phosphate buffer saline (PBS) three times. After removing the metaphysis, the bone marrow was flushed out and transferred to a 50 mL sterile centrifuge tube for centrifugation at 2,000 × g for 5 min. The obtained cells were seeded in DMEM and placed in an incubator for subculture. When cultured to the third passage, the cell surface antigens were detected using flow cytometry, and the qualified BMSCs were aliquoted and stored at −80°C for later use.

### 2.3. Extraction of BMSC Exosomal miR-146a

The BMSCs cultured to the third passage were seeded in a 10 cm cell culture dish, and the supernatant was obtained. Centrifugation (300 × g, 10 min) was then performed to remove the cells. The supernatant was then obtained and centrifuged for two times successively at a speed of 2,000 × g and 10,000 × g, respectively, with a centrifugation time of 10 min. The supernatant was extracted and centrifuged twice at 100,000 × g for 60 min. The obtained precipitate was retained, diluted with 200 *μ*L PBS solution, and stored at −80°C for later use.

RETRACTED

### 2.4. Establishment of a Mouse DR Model

Twenty-eight mice were randomly divided into a control group (*n* = 8) and an experimental group (*n* = 20); the former were fed basic feed and the latter were fed high-sugar and high-fat feed. After 8 weeks of feeding, all the experimental mice were fasted for 12 h. The experimental group was then injected with 60 mg/kg streptozotocin to produce a type 1 diabetic mouse model. The injection was continued for 5 d, and the blood glucose level of the mice was measured on the 7th day. A blood glucose level > 11.1 mmol/L indicated the successful establishment of the diabetic mouse model. Mice with successful diabetes modeling were normally fed for 4 weeks. After 4 weeks, telangiectasia, retinal hemorrhage, and arteriovenous abnormalities appeared in the fundus of the mice, indicating that the DR model was successfully constructed.

### 2.5. Preparation and Group Intervention of Microglias

The 16 DR mice were randomly separated into a model group and a miR-146a group, with 8 mice in each group. The retinal microglias of mice in each group were extracted. The DR mice were immersed in 75% alcohol for 10 min and then killed by rapid neck removal. The cerebral cortex of each animal was cut to remove the meninges and blood vessels. The obtained tissue was cut into pieces, and the suspension was obtained by pipetting and filtering with a sieve. The suspension was added to DMEM containing 10% PBS and placed in a constant temperature incubator for adherent culturing. When the culture reached the third passage, it was seeded in the culture flask, fixed, shaken at 250 × g on a constant temperature shaker for 30 min, and centrifuged (1,500 × g, 5 min) to collect the supernatant for inoculation into a 24-well plate. The miR-146a group was injected with 2.5 mg/kg of BMSC exosomal miR-146a, the model group was injected with saline (2.5 mg/kg), and the control group was not treated. pcDNA-CON and pcDNA-TLR4 were transfected into the DR mouse microglias and were set as the pcDNA-CON and pcDNA-TLR4 groups, respectively. Controlled plasmid (pcDNA 3.0) and pcDNA 3.0-TLR4 were obtained from Hanbio (Shanghai, China). After transfection of pcDNA-CON and pcDNA-TLR4, they were treated with BMSC exosomal miR-146a and were recorded as pcDNA − CON + miR − 146a group and pcDNA − TLR4 + miR − 146a groups, respectively.

RETRACTED

### 2.6. MTT Detection of Microglial Activity

The subcultured microglias were seeded in a 24-well vitreous plate and further cultured for 48 h. After two days, 20 *μ*L of MTT solution was added to each well for incubation. After incubating for 4 h, 150 *μ*L of DMSO was added to each well. The reaction was shaken for 10 min, and the absorbance was measured at 490 nm.

### 2.7. Detection of Microglial Apoptosis by Flow Cytometry

After the cells of different transfection groups were cultured for 48 h, they were rinsed twice with precooled PBS, resuspended in PBS binding buffer, and added with Annexin V-FITC (10 *μ*L) for 10 min of incubation. Five *μ*L of PI was added 10 min before cell apoptosis detection by flow cytometry.

### 2.8. Western Blot

The total protein content was extracted from cells using the radioimmunoprecipitation assay (RIPA) lysis buffer (Sigma, USA). After centrifugation, the protein samples were isolated from the supernatant. Protein concentration was determined by DC Protein Assay (BioRad, USA). Then, the obtained protein samples were electrophoresed and transferred to a membrane. After that, the membrane was incubated at 4°C for 12 h with the following primary antibodies: PCNA (1 *μ*g/ml, ab29, Abcam, UK), Bcl-2 (1 : 1000, ab32124, Abcam, UK), Bax (1 : 1000, ab32503, Abcam, UK), Caspase-3 (1 : 500, ab32042, Abcam, UK), TLR4 (1 : 1000, ab13556, Abcam, UK), MyD88 (1 : 1000, ab133739, Abcam, UK), NF-*κ*B (1 : 1000, ab288751, Abcam, UK), and *β*-actin (1 *μ*g/ml, ab8226, Abcam, UK). After washing the membrane with TBST, it was incubated with the HRP-labeled secondary antibody (1 : 2000, ab6721, Abcam, UK) at 37°C for 90 min. The membrane was washed with TBST and developed with an ECL luminescent solution. The gray value of the protein band was measured using the Quantity One software.

### 2.9. Serum TNF-*α*, IL-1*β*, and IL-6 Detection

The enzyme-linked immunosorbent assay method was used to detect the levels of TNF-*α*, IL-1*β*, and IL-6 in microglias. The specific steps are as follows: first, the specific antibody globulin was diluted with a coating buffer. The coating solution was then removed by 3 hours of immersion in a 37°C water bath as well as 3 times of rinsing with washing buffer. The test sample containing the antigen was added, and the enzyme-labeled specific antibody was added after incubation and washing. The substrate was added to develop color after another incubation and washing, and the results were observed.

### 2.10. Statistical Analysis

We used SPSS 23.0 to analyze the data of this study. All experiments were determined 3 times. Quantitative data conforming to a normal distribution are represented by mean ± standard deviation. Intergroup comparisons were performed using a one-way analysis of variance (ANOVA), and an SNA-Q was used for pairwise comparison between the two groups. For all data comparisons, we used a statistical significance level of *P* < 0.05.

RETRACTED

## 3. Results and Discussion

### 3.1. BMSC Identification

The results showed that the cell surface antigens CD29 and CD44 were positive, with the positive rates of 96.44% and 98.17%, respectively. CD31 and CD117 were negative. This indicated that the cultured cells were BMSCs. The results of the flow cytometry are shown in Figure 1.

### 3.2. Effects of BMSC Exosomal miR-146a on Microglial Proliferation

The ANOVA found that the level of proliferating cell antigen (PCNA) was significantly different among the three groups (*F* = 16.611, *P* < 0.05), which suggested that the proliferation rate of microglias in DR mice was higher than that in control mice. In microglias treated with BMSC exosomal miR-146a, the expression of PCNA and cell activity significantly decreased (*F* = 26.913, *P* < 0.05), as shown in Table 1 and Figure 2.

### 3.3. Effects of BMSC Exosomal miR-146a on Microglial Apoptosis

The ANOVA showed significantly different differences in the expression of Bax, Bcl-2, and Capase-3 and the apoptosis rate among the three groups (*P* < 0.05). Compared with the control group, the apoptosis rate of microglias and levels of Bax and Capase-3 in DR mice decreased significantly, while the levels of Bcl-2 significantly increased (*P* < 0.05). Following treatment with miR-146a, the apoptosis rate of microglias and levels of Bax and Capase-3 significantly increased, whereas the levels of Bcl-2 decreased (*P* < 0.05), as shown in Table 2 and Figures 3 and 4.

### 3.4. Effect of BMSC Exosomal miR-146a on TNF-*α*, IL-1*β*, and IL-6

We found that compared with untreated mice, the levels of TNF-*α*, IL-1*β*, and IL-6 in the microglias of DR mice treated with saline increased significantly (*P* < 0.05). However, after miR-146a treatment, these levels significantly decreased (*P* < 0.05), as shown in Table 3 and Figure 5.

### 3.5. Effects of BMSC Exosomal miR-146a on the TLR4/MyD88/NF-*κ*B Pathway

Compared with untreated mice, the expression of TLR4 in microglias of DR mice treated with saline significantly increased, and the activity of MyD88 and NF-*κ*B protein declined significantly (*P* < 0.05). After miR-146a treatment, the level of TLR4 in microglias significantly decreased, whereas the levels of MyD88 and NF-*κ*B proteins significantly increased (*P* < 0.05), as shown in Figure 6.

RETRACTED

### 3.6. Effect of PcDNA-TLR4 on Changes in Microglias Treated with miR-146a

Comparison with the pcDNA-CON group, the levels of PCNA and Bcl-2 in the pcDNA-TLR4 group significantly increased, and the levels of Bax and Capase-3 significantly decreased (*P* < 0.05). This showed that overexpression of TLR4 increased the proliferation ability and reduced the apoptosis ability of microglias. Compared with the pcDNA − CON + miR − 146a group, the PCNA and Bcl-2 levels of the pcDNA − TLR4 + miR − 146a group significantly increased, whereas the levels of Bax and Capase-3 decreased (*P* < 0.05). This suggested that overexpression of TLR4 reversed the effects of miR-146a on the proliferation and apoptosis of microglias, as shown in Table 4 and Figure 7.

### 3.7. Effect of PcDNA-TLR4 on the TLR4/MyD88/NF-*κ*B Pathway in Mice Treated with miR-146a

Compared with blank transfected cells, the TLR4 level of cells transfected with TLR4 was significantly increased, and the levels of MyD88 and NF-*κ*B both significantly decreased (*P* < 0.05). In comparison with the pcDNA − CON + miR − 146a group, the TLR4 level of the pcDNA − TLR4 + miR − 146a group increased significantly, whereas the levels of MyD88 and NF-*κ*B significantly decreased (*P* < 0.05), as shown in Table 5 and Figure 8.

## 4. Discussion

Diabetes affects more than 500 million adults worldwide and is a global public health issue. Studies have reported that about one third of diabetic patients experience varying degrees of vision loss or blindness due to DR [20]. Therefore, the treatment of DR is a focus of diabetes research. At present, the pathogenesis of DR is not yet fully understood, but it is believed to be related to the abnormality of the retinal microvascular system and is affected by a variety of factors [21, 22]. There is increasing evidence confirming that inflammation is a significant contributor to the development of DR [23–25]. DR patients are more prone to inflammatory reactions because of the high glucose environment in the body, which forms a vicious circle. During the development of DR, microglias are activated to proliferate and migrate, which can cause diabetic retinal neurodegeneration and microvascular circulation disorders [26]. A study found that in patients with DR, microglias accumulate in the injured nerve area and surround the new and expanded blood vessels, which aggravates the peripheral inflammation of microvessels [27]. Mesenchymal stem cell exosomes, which are naturally secreted nanoscale vesicles, have been shown to effectively reduce oxidative stress response and repair liver, kidney, and neuronal damage in patients with liver injury [28–30]. However, the mechanism of action of mesenchymal stem cell exosomes on microglias in DR patients remains poorly understood, and the application of exosomes in clinical treatment of DR is currently limited. Therefore, it is very important to deeply explore the mechanism of microglial apoptosis induced by BMSC exosomes, which can provide an experimental basis for the treatment of DR by exosomes.

RETRACTED

In this study, PCNA and Bcl-2 levels of microglias decreased following MBSC exosomal miR-146a treatment, while Bax and Capase-3 levels increased. Moreover, after miR-146a treatment, the levels of TNF-*α*, IL-1*β*, and IL-6 in microglias decreased. TNF-*α* is a small molecule protein secreted by macrophages, and its expression is regulated by the NF-*κ*B signaling pathway. Wang et al. showed that the levels of TNF-*α* in the tears of DR patients are proportional to the severity of the disease [31]. IL-1*β* is mainly produced by macrophages, which promotes the release of neutrophils from bone marrow and induces monocytes to release lysosomal enzymes locally, resulting in local inflammation. Animal studies have shown that injection of IL-1*β* into rat vitreous can cause degeneration of retinal capillary endothelial cells [32]. While IL-6, a multieffect factor with a wide range of functions, can regulate the growth of various cells and directly promote neovascularization [33]. Furthermore, IL-6 induces the formation of new blood vessels by promoting the secretion of vascular endothelial growth factor. Therefore, we suggest that miR-146a reduces the activation and proliferation of microglias and enhances apoptosis.

TLR4/MyD88/NF-*κ*B is a classical inflammation signaling pathway, which maintains the balance of inflammatory factors in the body. TLR4 can recognize the TLR4 receptors, respond quickly to danger signals that invade the body, and activate the pathway by binding to the TLR domain through MyD88 [34]. Numerous accumulated signal molecules are mediated by the IkB kinase complex, which phosphorylates IkB to lead to protease degradation. In turn, the NF-*κ*B dimer enters the nucleus and regulates the expression of target genes, thereby inducing inflammatory reactions [35]. Regulation of the TLR4/MyD88/NF-*κ*B pathway has been reported to decrease the release of inflammatory factors, thereby reducing the inflammatory response in colonic tissue [36]. In other rat experiments, stimulation of the TLR4/MyD88/NF-*κ*B pathway in the spinal cord promotes the production of IL-1*β* and TNF-*α*, which triggers an organ hypersensitivity reaction [37]. In this study, overexpression of TLR4 increased cell activity, enhanced proliferation, and decreased apoptosis. After treatment with miR-146a, the expression of TLR4 in microglias decreased, while the activity of MyD88 and NF-*κ*B increased, which indicated that miR-146a can reduce the activity of the TLR4/MyD88/NF-*κ*B pathway. Moreover, the overexpression of TLR4 reversed the effects of miR-146a on the proliferation and apoptosis of microglias and alleviated inflammation in DR mice.

RETRACTED

## 5. Conclusion

The number of activated microglias in the retina of DR mice increased significantly, which increased the release of inflammatory transmitters by microglias and exacerbated the damage to retinal blood vessels. After treatment with miR-146a, the proliferation ability of microglias decreased, the apoptosis increased, and the levels of inflammatory factors decreased. Further investigation found that overexpression of TLR4 enhanced cell proliferation, decreased apoptosis, and decreased the activity of MyD88 and NF-*κ*B. Furthermore, overexpression of TLR4 reversed the effects of miR-146a on microglia proliferation, apoptosis, and inflammation of DR mice. Therefore, this paper argues that BMSC exosomal miR-146a inhibits the proliferation of microglias by inhibiting the TLR4/MyD88/NF-*κ*B pathway, promoting apoptosis, and reducing the release of inflammatory factors, which ultimately reduces retinal damage.

## Figures and Tables

**Figure 1:** Detection of mesenchymal stem cells by flow cytometry. (a)–(d) Flow cytometry detects CD29, CD44, CD31, and CD117 surface antigens, respectively; *n* = 3.

**Figure 2:** Western blot detection of proliferating cell nuclear antigen (PCNA) protein levels. (a) Gray value of PCNA protein. (b) Relative expression of PCNA proteins. ^∗^ and # are comparisons with control and model groups, respectively; *P* < 0.05; *n* = 3.

**Figure 3:** Detection of microglial apoptosis by flow cytometry; *n* = 3.

**Figure 4:** Western blot detection of protein levels. (a) Gray value of proteins. (b) Relative protein expression of genes. ^∗^ and ^#^ are comparisons with control and model groups, respectively; *P* < 0.05; *n* = 3.

**Figure 5:** Expression of inflammatory factors. (a)–(c) Expression of TNF-*α*, IL-1*β*, and IL-6, respectively. ^∗^ and ^#^ are comparisons with control and model groups, respectively; *P* < 0.05; *n* = 3.

**Figure 6:** Western blot detection of protein levels. (a) Gray value of proteins. (b) Relative protein expression of genes. ^∗^ and ^#^ are comparisons with control and model groups, respectively; *P* < 0.05; *n* = 3.

**Figure 7:** Western blot detection of protein levels. (a) Gray value of proteins. (b) Relative protein expression of genes. ^∗^ and ^#^ are comparisons with pcDNA-CON and pcDNA − CON + miR − 146a groups, respectively; *P* < 0.05; *n* = 3.

RETRACTED

**Figure 8:** Western blot detection of TLR4, MyD88, and NF-*κ*B protein levels. (a) Gray value of TLR4, MyD88, and NF-*κ*B proteins. (b) Relative expression of TLR4, MyD88, and NF-*κ*B proteins. ^+^ and ^∗^ are comparisons with pcDNA-CON and pcDNA − CON + miR − 146a groups, respectively; *P* < 0.05; *n* = 3.

**Table 1:** miR-146a effects on microglial proliferation.

Group	PCNA	OD490 nm
Control	0.81 ± 0.13	0.61 ± 0.08
Model	1.26 ± 0.15^∗^	0.97 ± 0.12
miR-146a	0.96 ± 0.09^∗^#	0.79 ± 0.09
*F*	16.611	26.913
*P*	<0.001	<0.001

Note. ^∗^ and # are comparisons with the control and model groups, respectively; *P* < 0.05; *n* = 3.

**Table 2:** miR-146a effects on apoptosis of microglias.

Group	Bax	Bcl-2	Capase-3	Apoptosis rate (%)
Control	0.92 ± 0.08	0.51 ± 0.08	0.79 ± 0.06	29.34 ± 3.91
Model	0.69 ± 0.05^∗^	0.91 ± 0.11^#^	0.49 ± 0.07^#^	12.08 ± 2.47
miR-146a	0.81 ± 0.07^∗^^#^	0.74 ± 0.06^∗^^#^	0.61 ± 0.09^∗^^#^	21.08 ± 3.05
*F*	23.011	43.762	32.961	58.273
*P*	<0.001	<0.001	<0.001	<0.001

Note. a and b are comparisons with the control and model groups, respectively; *P* < 0.05.

**Table 3:** miR-146a effect on inflammatory factors (mean ± standard deviation).

Group	TNF-*α* (pg/mL)	IL-1*β* (pg/mL)	IL-6 (pg/mL)
Control	48.75 ± 7.95	11.97 ± 1.85	10.59 ± 2.28
Model	184.51 ± 32.08^∗^	32.71 ± 3.08^∗^	67.44 ± 9.85^∗^
miR-146a	106.17 ± 15.82^∗^^#^	19.64 ± 2.14^∗^^#^	31.08 ± 6.19^∗^^#^
*F*	83.022	203.514	141.632
*P*	<0.001	<0.001	<0.001

Note. a and b are comparisons with the control and model groups, respectively; *P* < 0.05; *n* = 3.

**Table 4:** pcDNA-TLR4 effects on miR-146a treated microglias.

Group	PCNA	Bax	Bcl-2	Capase-3
pcDNA-CON	0.89 ± 0.11	1.04 ± 0.11	0.93 ± 0.12	0.99 ± 0.13
pcDNA-TLR4	1.19 ± 0.13^∗^	0.67 ± 0.08^∗^	1.29 ± 0.15^∗^	0.61 ± 0.07^∗^
pcDNA − CON + miR − 146a	0.71 ± 0.09^∗^	1.23 ± 0.14^∗^	0.66 ± 0.08^∗^	1.25 ± 0.11^∗^
pcDNA − TLR4 + miR − 146a	1.02 ± 0.11^#^	0.82 ± 0.07^#^	0.81 ± 0.11^#^	0.76 ± 0.09^#^
*F*	26.814	45.003	41.722	59.501
*P*	<0.001	<0.001	<0.001	<0.001

Note. ^∗^ and # are comparisons with the pcDNA-CON and pcDNA − CON + miR − 146a groups, respectively; *P* < 0.05; *n* = 3.

**Table 5:** Effect of pcDNA-TLR4 on the TLR4/MyD88/NF-*κ*B pathway.

Group	TLR4	MyD88	NF-*κ*B
pcDNA-CON	0.91 ± 0.12	1.09 ± 0.11	1.12 ± 0.08
pcDNA-TLR4	1.25 ± 0.09^+^	0.71 ± 0.08^+^	0.74 ± 0.13^+^
pcDNA − CON + miR − 146a	0.69 ± 0.11^+^	1.21 ± 0.14^+^	1.18 ± 0.12^+^
pcDNA − TLR4 + miR − 146a	1.11 ± 0.14^∗^	0.93 ± 0.09^∗^	0.87 ± 0.11^∗^
*F*	35.114	32.393	86.591
*P*	<0.001	<0.001	<0.001

Note. ^+^ and ^∗^ are comparisons with the pcDNA-CON and pcDNA − CON + miR − 146a groups, respectively; *P* < 0.05; *n* = 3.

RETRACTED

## Data Availability

The simulation experiment data used to support the findings of this study are available from the corresponding author upon request.

## References

[1] Toprak I., Fenkci S. M., Fidan Yaylali G., Martin C., Yaylali V. (2020). Early retinal neurodegeneration in preclinical diabetic retinopathy: a multifactorial investigation. *Eye*.

[2] Cano J., O’neill W. D., Penn R. D. (2020). Classification of advanced and early stages of diabetic retinopathy from non-diabetic subjects by an ordinary least squares modeling method applied to octa images. *Biomedical Optics Express*.

[3] Yang M.-C., Zhu X.-B., Wang Y.-X. (2020). Influencing factors for peripheral and posterior lesions in mild non-proliferative diabetic retinopathy—the Kailuan eye study. *International Journal of Ophthalmology*.

[4] Khan A. A., Rahmani A. H., Aldebasi Y. H. (2018). Diabetic retinopathy: recent updates on different biomarkers and some therapeutic agents. *Current Diabetes Reviews*.

[5] Spencer B. G., Estevez J. J., Liu E., Craig J. E., Finnie J. W. (2020). Pericytes, inflammation, and diabetic retinopathy. *Inflammopharmacology*.

[6] Wang Y., Liu X., Zhu L. (2020). Pg545 alleviates diabetic retinopathy by promoting retinal Müller cell autophagy to inhibit the inflammatory response. *Biochemical and Biophysical Research Communications*.

[7] Li Y., Liu C., Wan X.-S., Li S.-W. (2018). Nlrp1 deficiency attenuates diabetic retinopathy (dr) in mice through suppressing inflammation response. *Biochemical and Biophysical Research Communications*.

[8] Liao Y.-R., Li Z.-J., Zeng P., Lan Y.-Q. (2017). Tlr7 deficiency contributes to attenuated diabetic retinopathy via inhibition of inflammatory response. *Biochemical and Biophysical Research Communications*.

[9] Zhu S.-H., Liu B.-Q., Hao M.-J. (2017). Paeoniflorin suppressed high glucose-induced retinal microglia mmp-9 expression and inflammatory response via inhibition of tlr4/nf-*κ*b pathway through upregulation of socs3 in diabetic retinopathy. *Inflammation*.

[10] Zhang T., Ouyang H., Mei X. (2019). Erianin alleviates diabetic retinopathy by reducing retinal inflammation initiated by microglial cellsviainhibiting hyperglycemia‐mediated ERK1/2–NF‐*κ*B signaling pathway. *The FASEB Journal*.

[11] Acuna L., Corbalán N. S., Raisman-Vozari R. (2020). Rifampicin quinone pretreatment improves neuronal survival by modulating microglia inflammation induced by *α*-synuclein. *Neural Regeneration Research*.

[12] Jian Y., Dong S., Xu S. (2020). Microrna-34a suppresses neuronal apoptosis and alleviates microglia inflammation by negatively targeting the notch pathway in spinal cord injury. *European Review for Medical and Pharmacological Sciences*.

RETRACTED

[13] Ji Y., Fang Q., Wang S. (2020). Lnc-rna blacat1 regulates differentiation of bone marrow stromal stem cells by targeting mir-142-5p in osteoarthritis. *European Review for Medical and Pharmacological Sciences*.

[14] Huan S., Jin J., Shi C., Li T., Dai Z., Fu X. (2020). Overexpression of mir-146a inhibits the apoptosis of hippocampal neurons of rats with cerebral hemorrhage by regulating autophagy. *Human & Experimental Toxicology*.

[15] Zhou Y., Zhou W., Chen X. (2020). Bone marrow mesenchymal stem cells-derived exosomes for penetrating and targeted chemotherapy of pancreatic cancer. *Acta Pharmaceutica Sinica B*.

[16] Yang H., Song X., Wei Z. (2020). Tlr4/myd88/nf-*κ*b signaling in the rostral ventrolateral medulla is involved in the depressor effect of candesartan in stress-induced hypertensive rats. *ACS Chemical Neuroscience*.

[17] Sun F., Liu F. (2020). Platycodin d inhibits mpp+-induced inflammatory response in bv-2 cells through the tlr4/myd88/nf-*κ*b signaling pathway. *Journal of Receptors and Signal Transduction*.

[18] Wei C.-B., Tao K., Jiang R., Zhou L.-D., Zhang Q.-H., Yuan C.-S. (2017). Quercetin protects mouse liver against triptolide-induced hepatic injury by restoring th17/treg balance through tim-3 and tlr4-myd88-nf-*κ*b pathway. *International Immunopharmacology*.

[19] Wang C., Yang Y.-H., Zhou L., Ding X.-L., Meng Y.-C., Han K. (2020). Curcumin alleviates ogd/r-induced pc12 cell damage via repressing ccl3 and inactivating tlr4/myd88/mapk/nf-*κ*b to suppress inflammation and apoptosis. *Journal of Pharmacy and Pharmacology*.

[20] Hou Y., Cai Y., Jia Z., Shi S. (2020). Risk factors and prevalence of diabetic retinopathy: a protocol for meta-analysis. *Medicine*.

[21] Chaurasia S. S., Lim R. R., Parikh B. H. (2018). The nlrp3 inflammasome may contribute to pathologic neovascularization in the advanced stages of diabetic retinopathy. *Scientific Reports*.

[22] Huang C., Zhu H., Li H. (2018). P38-mapk pathway is activated in retinopathy of microvascular disease of stz-induced diabetic rat model. *European Review for Medical and Pharmacological Sciences*.

[23] Qin Y. J., Chan S. O., Lin H. L. (2020). Increased expression of growth hormone–releasing hormone in fibrinous inflammation of proliferative diabetic retinopathy. *American Journal of Ophthalmology*.

[24] Xu K., Qian H., Zou M. (2020). Triamcinolone acetonide combined with aminoguanidine inhibits inflammation and oxidative stress, improves vascular endothelial and retinal function and reduces vegf expression in diabetic retinopathy patients. *Experimental and Therapeutic Medicine*.

[25] Qi F., Jiang X., Tong T., Chang H., Li R. (2020). mir-204 inhibits inflammation and cell apoptosis in retinopathy rats with diabetic retinopathy by regulating bcl-2 and sirt1 expressions. *European Review for Medical and Pharmacological Sciences*.

RETRACTED

[26] Ali S. A., Zaitone S. A., Dessouki A. A., Ali A. A. (2019). Pregabalin affords retinal neuroprotection in diabetic rats: suppression of retinal glutamate, microglia cell expression and apoptotic cell death. *Experimental Eye Research*.

[27] Grigsby J. G., Cardona S. M., Pouw C. E. (2014). The role of microglia in diabetic retinopathy. *Journal of Ophthalmology*.

[28] Wei X., Zheng W., Tian P. (2020). Administration of glycyrrhetinic acid reinforces therapeutic effects of mesenchymal stem cell-derived exosome against acute liver ischemia-reperfusion injury. *Journal of Cellular and Molecular Medicine*.

[29] Lee J. H., Shim Y. R., Seo W. (2020). Mitochondrial double-stranded rna in exosome promotes interleukin-17 production through toll-like receptor 3 in alcohol-associated liver injury. *Hepatology*.

[30] Zhang X.-W., Zhou J.-C., Peng D. (2020). Disrupting the trib3-sqstm1 interaction reduces liver fibrosis by restoring autophagy and suppressing exosome-mediated hsc activation. *Autophagy*.

[31] Wang T., Li J., Xie R. (2020). Intraocular tumour necrosis factor ligand related molecule 1 a links disease progression of proliferative diabetic retinopathy after primary vitrectomy. *Clinical and Experimental Pharmacology and Physiology*.

[32] Yao T. T., Yang Y., Jin X. L. (2020). Intraocular pharmacokinetics of anti-vascular endothelial growth factor agents by intraoperative subretinal versus intravitreal injection in silicone oil-filled eyes of proliferative diabetic retinopathy: a randomized controlled pilot study. *Acta Ophthalmologica*.

[33] Staszewski J., Skrobowska E., Piusińska-Macoch R., Brodacki B., Stępień A. (2019). Il-1*α* and il-6 predict vascular events or death in patients with cerebral small vessel disease—data from the shef-csvd study. *Advances in Medical Sciences*.

[34] Li Y., Xing N., Yuan J., Yang J. (2020). Sevoflurane attenuates cardiomyocyte apoptosis by mediating the mir-219a/aim2/tlr4/myd88 axis in myocardial ischemia/reperfusion injury in mice. *Cell Cycle*.

[35] Yuan S., Liu H., Yuan D. (2020). Pnpla3 i148m mediates the regulatory effect of nf-kb on inflammation in pa-treated hepg2 cells. *Journal of Cellular and Molecular Medicine*.

[36] Ye K., Chen Q. W., Sun Y. F., Lin J. A., Xu J. H. (2018). Loss of bmi-1 dampens migration and emt of colorectal cancer in inflammatory microenvironment through tlr4/md-2/myd88-mediated nf-*κ*b signaling. *Journal of Cellular Biochemistry*.

[37] Liu M., Xie J., Sun Y. (2020). Tlr4/myd88/nf-*κ*b-mediated inflammation contributes to cardiac dysfunction in rats of ptsd. *Cellular and Molecular Neurobiology*.

